RETRACTED

# A novel Skin lesion prediction and classification technique: ViT‐GradCAM

**DOI:** 10.1111/srt.70040

**Published:** 2024-09-02

**Authors:** Muhammad Shafiq, Kapil Aggarwal, Jagannathan Jayachandran, Gayathri Srinivasan, Rajasekhar Boddu, Adugna Alemayehu

**Affiliations:** ^1^ School of Information Engineering Qujing Normal University Qujing China; ^2^ Key Laboratory of Intelligent Sensor and System Design College of Information Engineering, Qujing Normal University Qujing China; ^3^ Department of CSE Koneru Lakshmaiah Education Foundation Vaddeswaram Andhra Pradesh India; ^4^ Department of Software and Systems Engineering School of Computer Science Engineering and Information Systems Vellore Institute of Technology, Katpadi Vellore India; ^5^ Department of Computer Science and Engineering Sathyabama Institute of Science and Technology Chennai India; ^6^ Department of AIML Gokaraju Rangaraju Institute of Engineering and Technology, Bachupally Hyderabad India; ^7^ Lecturer in Software Engineering Wachemo University Hosaina Ethiopia

**Keywords:** Grad‐CAM, linear patch projection, Multi‐Headed Self attention (MSA), multilayer perceptron (MLP), skin lesion, transformer encoder, vision transformer (ViT)

## Abstract

**Background:**

Skin cancer is one of the highly occurring diseases in human life. Early detection and treatment are the prime and necessary points to reduce the malignancy of infections. Deep learning techniques are supplementary tools to assist clinical experts in detecting and localizing skin lesions. Vision transformers (ViT) based on image segmentation classification using multiple classes provide fairly accurate detection and are gaining more popularity due to legitimate multiclass prediction capabilities.

**Materials and methods:**

In this research, we propose a new ViT Gradient‐Weighted Class Activation Mapping (GradCAM) based architecture named ViT‐GradCAM for detecting and classifying skin lesions by spreading ratio on the lesion's surface area. The proposed system is trained and validated using a HAM 10000 dataset by studying seven skin lesions. The database comprises 10 015 dermatoscopic images of varied sizes. The data preprocessing and data augmentation techniques are applied to overcome the class imbalance issues and improve the model's performance.

**Result:**

The proposed algorithm is based on ViT models that classify the dermatoscopic images into seven classes with an accuracy of 97.28%, precision of 98.51, recall of 95.2%, and an F1 score of 94.6, respectively. The proposed ViT‐GradCAM obtains better and more accurate detection and classification than other state‐of‐the‐art deep learning‐based skin lesion detection models. The architecture of ViT‐GradCAM is extensively visualized to highlight the actual pixels in essential regions associated with skin‐specific pathologies.

RETRACTED

**Conclusion:**

This research proposes an alternate solution to overcome the challenges of detecting and classifying skin lesions using ViTs and GradCAM, which play a significant role in detecting and classifying skin lesions accurately rather than relying solely on deep learning models.

## 1 INTRODUCTION

A skin lesion is an area of the skin with a different development pattern or texture from the surrounding skin. The primary and secondary skin lesions are the two types into which they can be separated. Primary skin lesions are abnormal skin conditions that may appear during childbirth or progress throughout an individual's life. Secondary skin lesions result from mistreated or irritated primary lesions. Granulation tissue, papules, tumors, and nodules are examples of first‐degree skin lesions; scales and ulcers are examples of secondary skin lesions. Malignant cancerous growths may sometimes be lethal.^1^ A severe kind of skin cancer is melanoma (MEL). One among the many severe skin malignancies brought on by aberrant skin growth of cells is malignant MEL, whose incidence has skyrocketed in the past few years. MEL, another name for cancerous tumors, originates at the melanocyte stage and extends to the top layers of the skin. The body's primary target regions, the face, neck, legs, and arms, are still exposed to sunlight. The World Health Organization (WHO) reports that more than three million other types of cancer diagnoses and over 132 000 occurrences of MEL are identified globally each year.^2^

Such severe disorder requires highly effective techniques to predict such classes. Medical pathologists can reduce disruptive noise and get outline data by accurately identifying the edge of the skin lesion.^3^ Deep learning has improved efficiency in analyzing images with an enormous amount of data with labels. However, because precise label generation necessitates specialist knowledge, acquiring pixel‐level annotation for identifying dermoscopic pictures is frequently costly. Various poorly supervised and semi‐supervised learning methods were recently put forth for categorization when there is little pixel‐level labeled information. Such methods enable precise classification using unlabeled or sparsely tagged information.^4^ Self‐learning is a semi‐supervised technique that generates artificial classifications to feed unlabeled samples by learning an instructional algorithm utilizing data with labels.

Moreover, complex challenges with learning that require assistance via conventional techniques based on rules can now be resolved thanks to deep learning. The efficiency of deep learning‐based algorithms on a range of complex computer vision and image classification assignments is almost on par with the abilities of humans. Therefore, deep‐learning algorithms are frequently used in healthcare imaging for various reasons, such as sickness diagnosis.^5^ Yet, deep structures must acquire many training cases to obtain valuable depictions. Creating extensive medical image datasets for supervised learning is more complicated than other applications. Purchasing and labeling are costly and time‐consuming, requiring specialized equipment and trained medical personnel. One of the main problems with contemporary deep learning and computer vision systems is data. There is insufficient data about skin conditions since many skin lesions and distinct characteristics exist.

RETRACTED

Due to such distinct characteristics, we proposed a novel classification and prediction technique called the ViT‐GradCAM model. We employed the vision transformer (ViT) technique to extract information from the images by converting it into the number of patches. Meanwhile, the deep learning model lacks visualization at the classification and some essential data loss in a fully connected network. To overcome this issue, Gradient‐Weighted Class Activation Mapping (GradCAM) is employed. The significant contribution of this proposal is listed as follows:

1. To employ primary data preprocessing and data augmentation to enrich the spatial feature extraction.
2. Class imbalance is minimized by generating artificial data to learn the proposed ViT‐GradCAM Technique better.
3. Augmentation of data with labels for better prediction of the spreading rate of skin lesions based on the class.
4. A gradient gradient‐weighted backpropagation process is carried out to avoid the loss of spatial information at the final layer.
5. To create a powerful, intuitive online tool that can identify and categorize skin lesions based on data collected in real‐time, helping medical professionals to receive an initial diagnosis.

The workflow of this framework is described as follows: Section 2 has the literature survey of some benchmarking skin disease classification techniques. Section 3 provides the methodology and mathematical model of the proposed ViT‐Grad CAM architecture. Section 4 shows the proposed model's proficiency by conducting experiments. The result shows that the proposed model outperforms other conventional classifying algorithms. Section 5 provides the conclusion of this framework.

## 2 RELATED WORKS

Zafar et al. (2023) proposed a ViT‐based skin lesion classification. In this paper, DeepLabv3+ model‐based segmentation of skin lesions is performed. Pretrained Mobilemetv2 is employed as the basic module of the DeepLabv3+ model. The feature map in the convolution layer is performed by the last convolution layer, which is the backbone of this network. As a result, the DeepLabv3+ model achieved an accuracy of 99.3% on the MED‐NODE dataset.^6^, ^18^ The ViTGAN‐based skin lesion classification was invented by Krishna et al. (2023). They employed a Generative adversarial network to perform data augmentation to resolve the class imbalance issue. Such intelligent skin classification techniques classified seven different classes of skin lesions using the HAM 10000 dataset. The experimental results show that the proposed model's training and testing accuracy achieved 99.2% and 97.4%, respectively.^7^, ^19^, ^20^, ^21^, ^22^, ^23^

Hao et al. (2023) proposed the ConvNeXt‐ST‐AFF model based on skin lesion classification. The proposed work concentrated on learning global features existing in the dataset image for better classification of lesions. The Swim ViT technique was integrated with the ConvNeXt model to strengthen the image classification. It enhanced the region of interest in the image to extract better features. The comparative analysis showed that the proposed model obtained an accuracy of about 92.16% while the precision, recall specificity, and f1 score were about 90.06%, 87.08%, 98.54%, and 88.83%, respectively.^8^ Stan et al. (2023) proposed the ViT model by introducing gradients at every stage; this method compels the model to identify the optimal features for our goal early.^9^, ^10^ In the subsequent example, we use a Kullback–Leibler divergence loss to push the consequent distribution of probabilities in line with one of the following levels, connecting the categorized heads of every successive level. The experimental results showed an accuracy of about 92.8% and a precision of about 91.53%, and the confusion matrix was generated to validate the proficiency of the proposed model.^11^

RETRACTED

Goseri et al. (2020) presented image augmentation techniques based on deep learning. It solves class imbalance and the image scarcity issue for training deep learning models. Moreover, the overfitting issue is discussed, and a solution for resolving the fitting problem is offered.^12^ Ayas (2022) presented the swim transformer model‐based classification of skin diseases. They focused on efficiently learning spatial data from the training images to enhance classification accuracy. As a result, reasonable outcomes were achieved by the presented model.^13^, ^14^, ^15^ However, it has certain drawbacks, detailed in Table 1.^14^

**TABLE 1:** Comparative analysis of existing skin lesion classification techniques.

Author	Year	Techniques	Results	Drawbacks
Zafar et al.^6^	2023	DeepLabv3+ model‐slim Mould Algorithm (SMA)	Achieved accuracy of about 99.3%	Lack of multiple classes classification of skin lesions
Krishna et al.^7^	2023	Lesion Aid ViT model	Achieved training accuracy of 99.2% and testing accuracy of 97.4%.	It's not a friendly model. It requires specific rules to be followed by the user to attain accurate results.
Hao et al.^8^	2023	ConvNeXt‐ST‐AFF model	Accuracy‐ 92.16% Precision‐ 90.06% Recall‐ 87.08% Specificity‐ 98.54% F1‐score‐ 88.83%	The primary constraint in this research is the heightened computing load caused by the model fusion methodology.
Stan et al.^11^	2023	Vision transformer	Accuracy‐ 92.8% Precision‐ 91.53% Recall‐ 86.73% F1‐score‐ 89.06%	Fails to classify all classes of skin lesions.
Goseri et al.^12^	2020	Survey of image augmentation techniques and overfitting elimination techniques based on deep learning	_	_
Arshed et al.^13^	2023	Vision transformer technique	Accuracy‐ 92.14% Precision‐ 92.61% Recall‐ 92.14% F1 score‐ 92.17%	Needs more enhancement in the preprocessing process.
Ayas S^14^	2022	Swim transformer model	Sensitivity‐ 82.3% Specificity‐ 97.9% Accuracy‐ 97.2% Balanced accuracy‐ 82.3%	Preprocessing and post‐processing stages were not integrated, degrading the model's classification performance.
Saha et al.^16^	2024	YoTransViT model	Accuracy of classification and precision of about 99.97% and 100%	Further investigation is to be implemented on more valuable datasets.
AISuwaidn L^17^	2023	Enhanced CNN model	Higher efficacy with an accuracy of 95.7%	More improvements in the presentation of readily available information from actual clinical trials and reliable machine‐learning diagnosis methods

## 3 METHODOLOGY

### 3.1 Overview

The primary goal of this study is to predict the skin lesion spreading rate and to classify the skin lesion under seven different classes, namely Actinic Ketratoses and intraepithelial carcinoma (AKIEC), Basal Cell Carcinoma (BCC), benign Keratosis lesions (BKL), dermatofibroma (DF), melanoma MEL, melanocytic nevi (NV), and vascular lesions (VASC). The overview of this research process is shown in Figure 1. The HAM 10000 dataset is selected to train and validate the proposed model. Due to class imbalance, data preprocessing and data augmentation have been done to overcome this issue. As a result, the number of samples from each class is enhanced, and the resultant sample is sufficient to train the ViT‐GradCAM model. After preprocessing and augmentation, the samples get fed to the transformer encoder, which generates the patch embedding and concatenates it with the tokens to enhance classification and prediction accuracy. At the final layer, the GradCAM technique is performed to extract the spatial features for visualization using the gradient weights generated by the backpropagation in the Grad‐CAM model. As a result, the spreading rate is evaluated based on the intensity of the patch and the actual class.

RETRACTED

**FIGURE 1:** Overview of ViD‐GradCAM.

### 3.2 Dataset

Human Against machine‐10 000 images (HAM 10000 dataset), one of the diverse datasets, has been chosen for training the proposed ViT‐GradCAM. https://www.kaggle.com/datasets/surajghuwalewala/ham1000‐segmentation‐and‐classification. The dataset has 10 015 images of skin lesions, which consist of seven different types of skin diseases, namely AKIEC, BCC, BKL, DF, MEL, NV, and VASC and the number of images in each class is about 327, 514, 1099, 115, 1113, 6705, and 142, respectively.^20^ Some of the sample images in the HAM 10000 dataset are shown in Figure 2. The diverse HAM 10000 dataset has high data imbalance in each class. To overcome this imbalance dataset, data augmentation is done in this research to generate the synthetic training images for better training of the proposed model. As a result of data augmentation, a wide number of images in each class are generated, which helps enhance classification accuracy. Table 2 depicts the dataset images under seven different classes.

**FIGURE 2:** Different skin lesion images in the HAM 10000 dataset.

**TABLE 2:** Different classes with a number of images in the HAM 10000 dataset.

Classes	Abbreviation	No. of images
Actinic keratoses and intraepithelial carcinoma	AKIEC	327
Basal Cell Carcinoma	BCC	514
Benign Keratosis‐like lesions	BKL	1099
Dermatofibroma	DF	115
Melanoma	MEL	1113
Melanocytic nevi	NV	6705
Vascular lesions	VASC	142

Abbreviations: AKIEC, Actinic Ketratoses and intraepithelial carcinoma; BCC, Basal Cell Carcinoma; BKL, benign Keratosis lesions; DF, dermatofibroma; MEL, melanoma; NV, melanocytic nevi; VASC, vascular lesions.

### 3.3 Data preprocessing and augmentation

#### 3.3.1 Data preprocessing

Data preprocessing is the crucial process for performance enhancement of machine learning models in image processing. It enhances the image quality by eliminating noise added to the training data. It removes the noise; thereby, the detection accuracy of ML models is improved. Generally, Preprocessing facilitates the effective extraction of target features from images and helps address problems like class in dataset imbalance, resulting in more reliable and accurate predictions. The HAM 10000 dataset consists of 10 015 images, which differ in size. To achieve consistency, all the images get resized into pixel size 224 × 224 without loss in disease‐affected regions.

RETRACTED

After resizing the image, its sharpness increases by removing the blurring effect. Here, the denoising filter removes the fading effect and the blurriness of skin lesion images in the HAM 10000 dataset. The Laplacian kernel operation is employed as a sharpening filter function. A Laplacian kernel with a positive core value encircled by negative values in a cross structure was applied to sharpen the data.

The Laplacian kernel function, that is, sharpening the Laplacian filter expression, is expressed in Equation (1).

(1) $$\Delta^{2}\;f_{l}=f_{l}\;\left(x+1,\;y\right)+f_{l}\left(x,y+1\right)+f_{l}\left(x-1,y\right)+f_{l}\left(x,y-1\right)-4f_{l}\left(x,y\right)$$

The sharpening Laplacian filter is well known for improving the edges of images and features despite preserving localized impacts and computing efficiency. However, because of its level of noise vulnerability, there is a chance that distortions may be introduced. Furthermore, the general aesthetic of a skin lesion image may be impacted by susceptibility to minor fluctuations and possible fringe impacts. When it applies to imaging for medical reasons, its usefulness depends on how carefully it is used, taking into account the amount of noise already present, to improve the sharpness of images for training the ViT‐GradCAM model. After preprocessing, we go on to the data augmentation process.

#### 3.3.2 Data augmentation

ViT models have been used widely in medical diagnostic applications for higher accuracy. The augmentation of the data on the training dataset images enhances such skillful framework performance. Here, the HAM 10000 dataset has diverse skin lesion images but has a high‐class imbalance, as shown in Figure 3. Basic augmentation operations such as flip (horizontal and vertical), shift, rotate, zoom (random), etc., are performed to overcome the imbalance issue.

**FIGURE 3:** Data augmentation process of HAM 10000 dataset images.

### 3.4 ViT‐GradCAM for skin lesion spreading rate prediction and classification

#### 3.4.1 Vision transformer mechanism

In general, the ViT method is one of the deep learning techniques. ViT uses a transformer to detect and classify the images in various applications. Especially in medical applications, accuracy is the main parameter for precisely detecting target regions in medical images. To achieve this goal, the ViT model is employed in this proposal to spread the rate of skin lesions over the patient's skin using the HAM 10000 dataset images, which are preprocessed and augmented. It has been demonstrated that ViT can produce cutting‐edge outcomes on several image identification targets, including Image Net. They are proficient in various image recognition tasks, such as scenarios and object identification. ViT performs exceptionally well but has a few improvements beyond other deep‐learning algorithms for classifying images. For instance, these algorithms need no human resizing or cropping when handling input photographs of any size, and they can be trained with comparatively minimal quantities of data; these qualities render them a viable option for image detection and classification in practical applications.

RETRACTED

ViT network uses a self‐attention mechanism to depict long‐range interdependence in the dataset image, which helps to enhance the spreading rate prediction accuracy and skin cancer classification accuracy. Instead of convolution layers in DL models, ViT uses a transformer encoder layer. The classification is performed using the transformer encoder, Multi‐Head Attention blocks, to enhance accurate feature extraction in the target region. Unlike traditional transformers, an input data image that can be reduced and converted into N patches is fed into the ViT architecture as a series of linear embedded data of the segregated patches.

As mentioned above, the transformer encoder in the ViT captures long‐range dependency in the number of patches fed into it. The number of segregated patches is named “tokens”. The number of patches/tokens generated is based on the below expression:

(2) $$N\;=\frac{h\;\times w}{p^{2}}\;$$

where N represents the number of tokens generated depending on the image pixel, handw represents the height and width of the actual image.

Steps of ViT to classify an image:

1. An image gets split into several patches.
2. Then, the patches get compressed into the linear patch using a feed‐forward layer called linear patch projection.
3. Then, the patches get converted into fixed vector size to produce the patch embedding.
4. The tokens are added with patch embedding for better classification of skin lesions.
5. After concatenating the embedding with tokens, the standard‐size vector tokens get fed to the transformer encoder.
6. The transformer encoder extracts the token sequence to classify the patches into corresponding classes.

The overview of the ViT is shown in Figure 4. The patch matrix is in the dimension of P,P which gets compressed into the dimension of $1,\;P^{2}$. The feed‐forward layer compresses the patch into a compressed matrix G. Then, the linear patch projection is produced in the dimension of $P^{2},\;F$. The patches get converted into an embedded patch $P_{e}$ with the fixed vector size F and the matrix dimension of patch embedding is 1,F. The Tokens are added with the patch embedding to feed the single input to the transformer encoder layer. Finally, the embedded patch $P_{e}$ gets added with the learnable token embedding $P_{el}$ which is considered a matrix concatenation, which resolves the issue $S_{class}$. The concatenated tokens get extracted using the expression.

(3) $$T_{o}=\;\left[S_{class};\;x_{1}\;P_{e};\;x_{2}\;P_{e};\text{…}\text{…}x_{n}\;P_{e}+\;P_{el}\right]$$

(4) $$P_{e}\in A^{F\times (P^{2}b)},P_{el}\;\in A^{F\times \left(N+1\right)}$$

**FIGURE 4:** Vision transformer.

RETRACTED

The transformer encoder consists of a multilayer MSA (multi‐headed self‐attention) block and an MLP (Multilayer Perceptron) block. The function of the transformer encoder is mathematically represented as

(5) $$T_{l^{,}}=\;MSA\left(LN\left(T_{l-1}\right)\right)+T_{l-1}$$

(6) $$T_{l}=\;MLP\left(LN\left(T_{l^{,}}\right)+T_{l^{,}}\right)$$

The MSA block performs a self‐attention (SA) mechanism, which is the key component in ViT. The SA extracts the key information from the image fed to the transformer encoder. Using the SA mechanism, a ViT model may focus on distinct areas of the input data according to their significance for the corresponding task. For this, the SA mechanism uses key, query, and value concepts. The key values get a dot product with query and are divided by the root of the dimension of the critical value, which is applied by a softmax function to get the weights. The concatenation of weights from the SA block is fed forward to the feed‐forward layer, which is expressed as,

(7) $$SA\;=W_{attention}\;\times V$$

(8) $$W_{attention}=\;softmax\left(QK^{T}\sqrt{K_{dim}}\right)$$

(9) $$MSA\;=\;concat\left(SA1,SA2,\;SA3,\text{…}\text{…}\text{…}.,\;SAn\right)\times W$$

(10) $$W\in A^{hK_{dim}\times F}$$

Then, the MLP block comprises two consecutive layers and a GELU activation function in between the successive layers. The basic function of MLP is to learn the complex information from the data. The complex data extraction in MLP is mathematically represented as

(11) $$MLP\;=\;GELU\left(XW_{1}+\;B_{1}\right)W_{2}+\;B_{2}$$

After extracting the class, the output of the transformer encoder gets passed to the final classification layer. In this research, based on the input data, we perform a GradCAM function for better accurate classification and spread rate prediction of skin lesions.

### 3.5 Gradient‐Weighted Class Activation Mapping (Grad‐CAM)

As in the case of deep learning networks, the final layer neurons consist of spatial information in the image for better detection and classification. Unfortunately, some essential spatial information lasts in FC layers in DL networks. To overcome this issue, Grad‐CAM is employed in this research at the final layer of the ViT. Grad‐CAM assigns fundamental values to every neuron in the final layer using gradient information. In this section, the output layer function is concentrated to explain the function of the final layer.

RETRACTED

For each class of width W and height H, the Grad‐CAM belongs to width and height, which is represented as

(12) $$L_{Grad-CAM}^{C}\in R^{W\times H}$$

The localization map with a discriminative class is obtained by calculating the backpropagation gradient value for each class based on the activation map features. $A^{k}$ that is $\frac{\;\partial x^{c}}{\partial {A^{k}}_{mn}}$. The backpropagation of weights having width and height is indexed with m and n, respectively, to get the weight of essential neuron in the final layer $\sigma_{c}$.

(13) $$\propto_{c}=\frac{1}{Z}\;\sum_{m}\sum_{n}\frac{\;\partial x^{c}}{\partial {A^{k}}_{mn}}$$

The weighted combination of activation map followed by ReLU activation mapping is done to obtain the average gradient value to obtain the matrix using the expression 14. The corresponding matrix gets combined with the actual image to represent spatial features.

(14) $$L_{Grad-CAM}^{c}=\;ReLU\left(\sum_{k}\propto_{c}A^{k}\right)$$

Here, we employ ReLU activation to the linear combination of weighted maps. Hence, we have to predict the spreading rate of the lesion over the skin, which depends upon the class, that is, the features having the infected region (positive), the intensity of a pixel is high $x^{c}$ when compared with the average skin pixel intensity. The negative pixel represents normal skin. Meanwhile, no ReLU prediction is less accurate and results in an inaccurate prediction rate.

**Table:** 

**Pseudo code**:
// Vision transformer ViT (input) Patch = create patch (input) Patch embedding = patch embedding (patch) Linear Sequence = concat (token, patch embedding) + position embedding Hidden state = transformer (linear sequence) Class‐output = calss head (hiddenstate) // Gradient‐Weighted Class Activation Mapping Class k, class head *N* Optimize (*N*) = select (Class head) Decompose‐feature (threshold ∝) For (*i* = 1,2,….,N) Calculate = CAM (Equation 13) Select = nearest (grad weight) for *k* in {*k*} do Calculate = $L_{Grad-CAM}^{c}$ (Equation 14) End for Patch $N(1+N_{con})$ instances from class head End for Return class output

## 4 RESULTS AND DISCUSSION

The performance of the proposed VIT‐Grad CAM technique is analyzed in this section. As a result, the proposed model achieved a prediction and classification accuracy of about 96.6%, which is comparatively higher than other conventional techniques. The confusion matrix visualizes the accurate classification of the ViT‐GradCAM model under seven different classes.

RETRACTED

### 4.1 Experimental setup

The experiment is done on the Windows 10 operating system with an i9 11th generation core processor and Nvidia RTX 3070 Ti GPU, a superior performance GPU, to train and test the proposed ViT GradCAM model. The Python 3.9 framework was constructed using Pytorch, Tensorflow 2.0, Keras, and OpenCV modules.

### 4.2 Evaluation metrics

Evaluation metrics are one of the important factors in analyzing the performance of any deep learning model. Based on the evaluation metrics percentage, the proposed model validated whether it performs well. Hence, we considered four evaluation metrics to validate the performance of the proposed model ViT‐GradCAM. The explanation and expression for these four parameters are detailed as follows.

1. **Accuracy** is the ratio of correctly identified images to the total number of images. Based on the accuracy, the overall performance of the proposed model is validated.
(15) $$Accuracy\;=\frac{TP+TN}{TP+TN+FP+FN}\;$$
2. **Precision**: It is the measure of accurate positive prediction. It is the ratio of true positive images, that is, images under appropriate skin lesion class, to the sum of true positive and false positives.
(16) $$Precision\;=\frac{TP}{TP+FP}\;$$
3. **Recall**: It measures identifying the positive images over all the positive images. It is the ratio of true positive images identified to the sum of true positive and false negative images.
(17) $$Recall\;=\frac{TP}{TP+FN}\;$$
4. **F1‐Score**: It is the harmonic average of precision and recall. It is helpful when there is an unequal distribution of classes or a comparable focus on both types of errors since it offers a single statistic that combines recall and precision.
(18) $$F1score\;=\;2\times \frac{Precisoin\times recall}{precision+recall}$$

The ratio of accurate predictions (true positives and negatives) to all projections, irrespective of class, is used to calculate efficiency in classifications with multiple courses. Comparatively, accuracy, recall, and F1 have considered gradient‐weighed values for multiple courses. Using gradient‐weighted values, each class's relative importance in data collection is determined by its proportion. The recall, accuracy, and score of F1 for every class are increased by the relevant gradient weights to create balanced weight metrics. The results are subsequently added up and divided by the total weight.

### 4.3 Performance analysis

This proposal considers the skin lesion classification and spreading rate prediction analysis. To validate the efficacy of the proposed ViT‐GramCAM model, some parameters are considered to visualize the state‐of‐the‐art performance of skin lesion prediction. The deep learning model performance is generally based on the learning rate while training and testing the data. Our proposed ViT‐GradCAM model achieved 96.6% accuracy at a learning rate of 0.6, as shown in Figure 5. While increasing the learning rate from 0.2 to 0.6, the prediction accuracy gets enhanced. Here, we compared the two techniques to validate the proposed model: The ViT technique^13^ and YoTransViT.^16^

RETRACTED

**FIGURE 5:** (A) and (B) accuracy and loss analysis of the proposed method.

In this analysis, we considered prediction accuracy from the images fed to the transformer encoder layer. The proposed ViT‐GradCAM model analyzed and processed the path embedding and extracts token sand spatial features from the embedding to classify skin lesions. As a result, the accuracy of the ViT‐GradCAM model achieved 96.6%, as shown in Figure 5A. The accuracy of the ViT technique is lower than that of the proposed Yo TransViT technique. Due to the GradCAM, the loss of information in a fully connected layer gets reduced. So, the prediction accuracy gets enhanced.

Meanwhile, the loss percentage is analyzed to determine the proficiency of the proposed model. The loss analysis graph is shown in Figure 5B. The loss gets reduced when the number of epochs increases. Based on the learning rate, the loss gets diminished. Here, the loss percentage is less for the proposed ViT‐GradCAM model when compared with the other two models.

The performance validation of ViT‐GradCAM is done by comparing the testing and training loss, as shown in Figure 6A. Then, the test and training accuracy is shown in Figure 6B. Figure 6A depicts that the loss decreases while the number of Epochs increases. Meanwhile, Figure 6B shows that the prediction accuracy gets enhanced by increasing the number of epochs. As a result, the prediction of the spreading rate for each sample gets enhanced. The categorization approach faces many difficulties because images in the seven classes appear identical. Even though skin lesion prediction and classification have been the subject of multiple published research, the suggested model's stability was more precise.

**FIGURE 6:** (A) Training loss versus test loss. (B) Training accuracy versus test accuracy using ViT‐GradCAM.

Understanding how DL techniques perform throughout training requires understanding learning diagrams representing the testing and training mechanisms. The graphs we create then allow us to keep an eye on and evaluate the performance that results from the framework, identify any overfitting problems, modify the structure of the ViT‐GradCAM model and hyperparameters as needed, and eventually improve the proposed model's accuracy and dependability. An illustration of the learning graphs visually is shown in Figure 7 at different learning rates. While increasing the learning rate from 0.2 to 0.6, prediction accuracy is enhanced by up to 15%.

RETRACTED

**FIGURE 7:** Accuracy analysis at different learning rates 0.6, 0.4, and 0.2.

The analysis of the spreading rate of lesions over the skin is based on the intensity of the gradient value generated by the ViT‐GradCAM model. The spreading rate prediction based on the intensity is shown in Figure 8. The graph shows that the spreading rate increases linearly with increased intensity. If the pixel's intensity is high, the spreading rate becomes severe; hence, immediate diagnosis is required. If the intensity is less, the spreading rate will become less. This indicates that the proposed model predicts the image more accurately based on the intensity of the pixels in the image.

**FIGURE 8:** Intensity versus spreading rate.

Then, the classification accuracy is validated by generating the confusion matrix. The confusion matrix can help evaluate a model's classification efficacy. At the same time, there are numerous uneven classes, and incorrectly categorizing a single category would result in a lot instead of misclassifying a different one. The accuracy, precision, recall, and F1 score parameters can be obtained from a confusion matrix.

In Figure 9, we consider 150 samples to test the classification efficacy of the proposed ViT‐GradCAM model. Twenty samples in the AKIEC class, 23 samples from DF, and the rest of the classes are shown in Table 3.

**FIGURE 9:** Confusion matrix of class prediction using ViT‐GradCAM.

**TABLE 3:** Number of images under seven different classes.

No. of samples	AKIEC	BCC	BKL	DF	MEL	NV	VASC
150	20	30	25	23	22	18	12

Abbreviations: AKIEC, Actinic Ketratoses and intraepithelial carcinoma; BCC, Basal Cell Carcinoma; BKL, benign Keratosis lesions; DF, dermatofibroma; MEL, melanoma; NV, melanocytic nevi; VASC, vascular lesions.

The average accuracy of classification under every class achieved about 97.2% approximately. The comparative analysis of accuracy, precision, recall, and F1score is discussed in the following subsection.

### 4.4 Comparative analysis

The proposed ViT‐GradCAM model is compared with three benchmarking models such as CNN‐based classification of the dermatological disorder,^17^ ViT‐based skin lesion generation, and classification,^13^ and YoTransViT‐based skin disease classification.^16^ The comparative results depict that the proposed ViT‐GradCAM achieved higher order accuracy of about 97.2%, the precision of about 98.5%, recall of about 95.5%, and F1 score of about 94.6%. YoTransViT model achieved the second highest accuracy, and the CNN model achieved the lowest accuracy due to the loss of essential spatial information in the fully connected layer shown in Figure 10. The overall comparison outcomes are listed in Table 4. As in the proposed model, the GradCAM effectively retains spatial information and back‐propagates it to the classification layer, and the appropriate class gets classified accurately.

RETRACTED

**FIGURE 10:** A comparative analysis of different deep learning models.

**TABLE 4:** Overall comparative analysis of Skin disease classification techniques.

Authors	technique	Evaluation metric	outcomes
Aisuwaidan et al.^17^	CNN‐based classification of dermatological disorder	Accuracy	91.1%
		Precision	90.3%
		Recall	92.4%
		F1 score	91.2%
Arshed et al.^13^	ViT‐based skin lesion classification	Accuracy	92.14%
		Precision	92.61%
		Recall	92.14%
		F1 score	92.17%
Saha et al.^16^	YoTrans Vit‐based skin disease classification	Accuracy	96.97%
Proposed	ViT‐GradCAM‐based skin lesion prediction and classification	Accuracy	97.28%
		Precision	98.51%
		Recall	95.2%
		F1 score	94.6%

## 5 CONCLUSION

The classification of skin lesions under seven different categories becomes challenging because of the high similarity index among all the categories. The primary identification method is visual, commencing with medical screening and progressing through dermoscopic analysis, histopathological evaluation, and specimen acquisition. Deep learning approaches accomplish significantly separated and presumably ubiquitous activities when applied to a categorized extremely fine object. This proposal proposes a novel ViT technique that integrates the Gradient‐weight activation mapping method for spreading rate prediction and classification of skin lesions. As a result, the proposed ViT‐GradCAM model accurately classified the images under seven categories with 97.28% accuracy. Compared with other DL techniques, our proposed model performance is enhanced. GradCAM is a method for seeing the input patch and applying the ViT framework to anticipate the lesion. The overall precision, recall, and F1score achieved by the proposed model are 98.51%, 95.2%, and 94.6%, respectively. The experimental results show the state‐of‐the‐art performance of the proposed ViT‐GradCAM technique.

## CONFLICT OF INTEREST STATEMENT

The authors declare no conflicts of interest.

## ETHICS STATEMENT

This study does not report on or involve any animals, humans, human tissue, or plants. Therefore, ethical approval and consent to participate were not required for this research. Informed consent was obtained from all authors for participation in this study and publication of the resulting manuscript.

RETRACTED

## Data Availability

The data that support the findings of this study are available from the corresponding author upon reasonable request.
